# HIV testing in jails: Comparing strategies to maximize engagement in HIV treatment and prevention

**DOI:** 10.1371/journal.pone.0286805

**Published:** 2023-06-23

**Authors:** Samantha R. Levano, Mallory E. Epting, Jacob A. Pluznik, Victoria Philips, Lindsey R. Riback, Chenshu Zhang, Binyam Aseffa, Aman R. Kapadia, Chava J. Bowden, Beth Jordan, Eleni O’Donovan, Anne C. Spaulding, Matthew J. Akiyama

**Affiliations:** 1 Department of Epidemiology, Rollins School of Public Health, Emory University, Atlanta, Georgia, United States of America; 2 Divisions of General Internal Medicine & Infectious Diseases, Montefiore Medical Center, Albert Einstein College of Medicine, Bronx, New York, United States of America; 3 D.C Department of Corrections, Washington, D.C., United States of America; 4 Unity Health Care, Washington, D.C., United States of America; Yale School of Medicine, UNITED STATES

## Abstract

Despite 15,000 people enter US jails yearly with undiagnosed HIV infection, routine HIV testing is not standard. Maximizing the yield and speed of HIV testing in short-term detention facilities could promote rapid entry or re-entry of people living with HIV (PLWH) into care. The goal of this study was to evaluate the impact of third generation, rapid point-of-care (rPOC) vs. fourth generation, laboratory-based antigen/antibody (LBAg/Ab) testing on the HIV care cascade in a large urban jail during a planned transition. We used aggregate historical data to compare rPOC testing and LBAg/Ab testing in the D.C. Department of Corrections. We examined two time periods, January to August 2019 when rPOC testing was performed, and October 2019 to January 2020 after LBAg/Ab testing began. We calculated monthly rates of HIV tests performed, HIV test results received, HIV test results received among those tested, antiretroviral therapy (ART) initiation, and proportion of PLWH receiving discharge planning prior to release. We then conducted an interrupted time series analysis to assess the differences between testing periods. There were 14,237 entrants during the first time period and 7,569 entrants during the second. Transitioning from rPOC to LBAg/Ab testing increased the rate of test uptake by 38.5% (95% CI: 14.0, 68.3), decreased the rate of test results received among those tested by 13.1% (95% CI: -14.0, -12.1), and increased the combined rate of HIV tests performed and results received by 20.4% (95% CI: 1.5, 42.8). Although the rate of HIV testing was greater under LBAg/Ab, PLWH received results immediately through rPOC testing, which is critically important in short-stay enviroments. Increasing rPOC uptake would increase its value and combined testing may maximize the detection of HIV and receipt of results among persons passing through jails.

## Introduction

Correctional settings, comprising in the United States (U.S.) prisons and jails, had a prevalence of 1.3% of people living with HIV (PLWH) in December 2015 [1]. With 10.9 million correctional admissions over the year, representing 7.8 million individuals since jail entrants enter on average 1.4 times annually, this translates to likely 100,000 PLWH incarcerated in the U.S. in 2015 [2, 3]. The correctional HIV epidemic encompasses a diverse group of individuals with varying levels of disease awareness, ability to manage their disease due to active substance use disorders, and care engagement [3].

Screening upon incarceration is warranted as it improves the positioning of PLWH in the HIV care continuum [4, 5]. Those knowledgeable about their HIV status and on antiretroviral therapy (ART) risk interruptions unless jail health care staff are alerted to the diagnosis. It provides the opportunity to initiate treatment for those known to be positive, but not linked to care, and identify those yet to be diagnosed. The latter group is of particular interest as a meta-analysis indicated that up to 15% of individuals entering corrections have undiagnosed HIV infections [6]. A survey of imprisoned people, conducted less than a year after prison officials reported 1.3% of persons were infected, found that 1.1% (or 15% less than 1.3%) reported they were PLWH [1, 7]. We estimate that 15,000 PLWH enter U.S. correctional facilities each year unaware of their HIV status.

The division of the U.S. correctional system into prisons and jails has implications for optimal screening strategies. In prisons, sentences are typically greater than one year whereas jails are shorter-term facilities with lengths of stay that can be unpredictable, ranging from just several hours to months depending on whether a resident is awaiting trial for a misdemeanor or felony, or has received a short sentence [3, 8]. Jails are the most common entry point into the correctional system and admissions to U.S. jails number approximately eighteen times the entrances in state and federal prisons [1, 3, 9–11]. About 95% of persons who leave the carceral environment have only been in jails [3]. Due to the high volume of PLWH cycling through these facilities, engagement with jails is essential to ending the HIV epidemic in the U.S.

Although testing for HIV in jails can be a critical step in improving health outcomes for PLWH and reducing the risk of transmission after release, routine testing is not the norm in U.S. jails [9, 10]. The recommendations of the Centers for Disease Control and Prevention (CDC) have focused on universal, opt-out testing as a diagnostic strategy for PLWH in correctional facilities. The CDC endorses rapid point-of-care testing (rPOC) in the jail setting, which has been found to be feasible and acceptable, followed by confirmatory laboratory-based testing [11–13]. Conventional laboratory-based HIV testing has higher specificity, and higher sensitivity than rPOC. Due to its higher sensitivity, especially in early disease, fourth generation laboratory-based antigen/antibody (LBAg/Ab) testing may identify patients with acute HIV infection, when rPOC would be falsely negative. Yet, because both rPOC and LBAg/Ab can yield false positive results if used alone, an additional HIV RNA viral load assay is recommended, which adds more time to receive final diagnostic results [14]. Laboratory testing alone may be acceptable for prisons, when turnaround time is not an issue [15]. However, when detained populations turnover swiftly in jails, rPOC testing may lead to the highest proportion of entrants, including undiagnosed PLWH, accessing test results before release [8, 16]. Because of short lengths of stay in jails, rPOC HIV testing potentially offer the greatest chance to identify in a timely manner cases previously undiagnosed, who may subsequently be linked to care.

In September 2019, the Washington, D.C. Department of Health (DOH) recommended a transition from rPOC to LBAg/Ab testing, which would be done in conjunction with a battery of other blood tests drawn at intake, as a strategy to find more cases of acute HIV. Unity Healthcare (UHC), the largest network of Federally Qualified Health Centers in D.C., has contracted to provide healthcare for the D.C. DOC since 2006. The Washington D.C. Department of Corrections (DOC), DOH, and UHC agreed to utilize this transition as a critical opportunity to study optimal HIV testing strategies in the jail setting. The goal of this study was to compare the rates of HIV tests performed, HIV test results received, ART initiated, and the ratio of PLWH receiving discharge planning prior to release under each testing strategy.

## Materials and methods

### Setting

The D.C. correctional system consists of single large urban jail, which ranks among the top 50 largest jails in the U.S. [17]. Prior to the COVID-19 pandemic, the D.C. DOC processed 6,000 to 8,000 intakes per year and housed an average daily population of approximately 1,800 individuals. The demographic distribution of the patient population is over 90% African American, 5% Latinx, and 3% White. Nearly all entrants live at or below the 200% poverty level. Approximately 92% of intakes are persons born male, with a male median age of 33 years and a female median age of 37 years. About 55% of patients have a history of substance abuse, mental illness, or both. The median length of stay in the D.C. DOC is 24 days for men and 13 days for women; 36% are released within 8 days of admission [18].

The HIV prevalence in the jail ranges from 1–2%, with an average estimated population of approximately 30 PLWH at any given time before the COVID-19 pandemic. In 2006, the D.C. DOC began routinely offering opt-out rPOC testing at entry. Initially, UHC made 1–3 novel HIV diagnoses in the jail each month through the rPOC HIV testing strategy, but in recent years these numbers began to fall (Personal communication–Ms. T. Outlaw, October 4, 2021).

At intake, UHC notifies entrants that they routinely test nearly all patients for HIV, at which time persons are able to decline or defer testing. Entrants who are known to be living with HIV, either through self-identification or a previous stay, are usually not re-offered HIV testing. Those tested within the last 6 months at the D.C. DOC are also not routinely retested.

Immediately before HIV testing transitioned to the laboratory-based strategy, medical assistants performed rPOC using a 1-minute INSTI HIV-1/HIV-2 Antibody Test (bioLytical Laboratories, Vancouver BC). Under LBAg/Ab, the fourth generation Architect HIV Ag/Ab Combo assay (Abbott Laboratories, Abbott Park, IL) was added to a larger infectious disease screening panel. Routinely at the jail, all laboratory-based test results are disseminated to patients based on their disease status. Individuals whose laboratory-based HIV tests were negative receive a letter in jail indicating that their intake laboratory results were normal. HIV testing is not mentioned specifically in this letter for confidentiality purposes. Individuals whose laboratory-based HIV tests were positive are notified of their results through a clinical, urgent care, or sick call visit scheduled within 24 hours of the laboratory result processing. A comprehensive clinical visit is then scheduled within two weeks for those who tested HIV positive at intake. For those already released, a letter is sent to the patient’s address on file, if one exists.

## Analysis

In this retrospective cohort study, we used aggregate historical data provided by the D.C. DOC and UHC to examine two study periods: January 2019 to August 2019 and October 2019 to January 2020, before the COVID-19 epidemic prompted decarceration. The D.C. DOC performed third generation, rPOC testing during the first period and fourth generation, LBAg/Ab testing in the second period. Because the transition in testing occurred part-way through September 2019, we designated this month as a washout period. The aggregate data from each time period included the total numbers and monthly averages as applicable for the following variables: jail admissions; HIV tests performed; HIV positive test results; entrants receiving positive and negative HIV test results; PLWH who received ART while in jail; discharge planning visits received by PLWH prior to release; PLWH released. We then calculated the monthly rate of tests performed, result received, tests performed and results received combined, ART initiation, and ratio of discharge planning visits to PLWH released per month across each time period. The total number of entrants receiving HIV test results was assumed to be 100% in the first time period since rPOC results for the test used were available in one minute from the point where care was delivered; however, we also conducted a sensitivity analysis by comparing just the receipt of results through the total number of letters generated for tests performed at intake in both the first and second time periods.

We compared the averages for each time period using two independent sample t-tests with a 5% critical level of significance. We then conducted an interrupted time series (ITS) analysis to assess the significance of the difference between each testing phase using negative binomial models. We calculated IRR (incidence rate ratio), which was expressed as a rate change in percentage between the two testing phases. Additionally, we assessed possible time trends within each testing period.

The Emory University Institutional Review Board approved our study. Data provided by the DOC were de-identified and presented as aggregate counts of study participants per month. Participants were not able to opt out of the study given the retrospective cohort design; therefore, a waiver of consent was obtained. Participants were, however, able to opt out of routine rPOC and LBAg/Ab testing at intake, which would lead to their data not being included in the study data set. There was no benefit or treatment associated with the data transfer for those whose data are included in the study.

## Results

The analysis included 6,075 entrants (67.4% of our study population) during the first time period and 2,941 entrants (32.6% of our study population) during the second (Table 1). Among the jail entrants during the first time period, 4,012 rPOC tests were performed (an average of 501.5 rPOC tests per month) (Table 1). All entrants (100%) were assumed to have received their rPOC HIV test results due to the nature of the rapid testing strategy; 410 (an average of 51.3 persons per month) PLWH were treated for HIV infection at the beginning of each month (Table 1). Additionally, 284 discharge planning visits (an average of 35.5 visits per month) were conducted with PLWH prior to release (Table 1). After the transition to LBAg/Ab testing, the D.C. DOC reported that 2,601 HIV tests were performed (an average of 650.3 LBAg/Ab tests per month) among the 2,941 jail entrants (Table 1). Approximately 2,282 entrants total received their HIV results, whether positive or negative (Table 1). Across this time period, 251 (an average of 62.8 persons per month) PLWH were treated for HIV infection at the beginning of each month (Table 1). Lastly, a total of 119 discharge planning visits (an average of 29.8 visits per month) were conducted with PLWH prior to release (Table 1).

**Table 1:** Descriptive statistics of HIV care and treatment outcomes in the D.C. DOC per month.

Variable	Rapid Point-of-Care Period (January 2019-August 2019)	Laboratory-Based Antigen/Antibody Period (October 2019-January 2020)
	Mean [Standard Deviation]	
Total Jail Entrants per Month	759.4 [22.2]	735.3 [10.8]
HIV Tests Performed per Month	548.4 [44.4]	651.0 [22.3]
Total Results Received per Month	518.9 [57.7]	570.5 [21.4]
Number of PLWH Receiving ARV on First of the Month	51.3 [5.8]	62.8 [4.8]
PLWH Released per Month	20.5 [3.7]	18.8 [3.6]
PLWH Received Discharge Planning Visit	35.5 [5.7]	29.8 [5.0]

The interrupted times series analysis demonstrated that, among those engaged in rPOC testing, the rate of performing an HIV test was 64.7% in August 2019 (95% CI: 55.8, 75.0); there was no change observed in the testing rate across the the rPOC testing period (Table 2). After the transition to LBAg/Ab testing, the rate of performing an HIV test significantly increased by 38.5 (95% CI: 14.0, 68.3) to 89.6% (Baseline* (1+Transition Change); the testing rate did not change across the LBAg/Ab testing period (Fig 1, Table 2). Regarding the receipt of test results, the predicted probability of receiving rPOC results was 100.0%; this baseline rate was assumed for the rPOC testing period. After the transition to LBAg/Ab testing, the predicted probability of receiving LBAg/Ab results started at 86.9% (95% CI: -14.0, -12.1) and then increased significantly by 0.6% from the new baseline in each following month (95% CI: 0.3, 1.0) (Fig 1, Table 2). This difference between testing periods was statistically significant in both the analysis where we assumed that 100% received rPOC test results and the sensitivity analysis of relying only on notifications generated for tests performed at intake (sensitivity analysis not shown). The rate of both performing an HIV test and receiving an HIV test result was 64.7% in August 2019 (95% CI: 56.8, 73.6) (Table 2). There was no significant change in the combined rate across the the rPOC testing period. The rate of performing an HIV test and receiving an HIV test result significantly increased to 77.9% (95% CI: 1.5, 42.8) after the transition to LBAg/Ab testing (Fig 1, Table 2); the testing rate did not change across the LBAg/Ab testing period.

**Fig 1:** Total number of entrants and rate of HIV testing and results received, Washington D.C. Department of Corrections jail, 2019–2020.

**Table 2:** Level and trend changes in predicted rates^a^ in HIV care and treatment.

	Rapid Point-of-Care Period (January 2019-August 2019)		Laboratory-Based Antigen/Antibody Period (October 2019-January 2020)	
	Baseline^b^ (%) (95% CI; p-value)	Pre-Transition Trend^c^ (Δ%) (95% CI)	Transition Change^d^ (%) (95% CI)	Post-Transition Trend^e^ (Δ%) (95% CI)
Rate of HIV Tests Performed	64.7 (55.8, 75.0)	-0.4 (-2.8, 2.1)	38.5 (14.0, 68.3)	-0.9 (-7.3, 6.1)
Rate of HIV Test Results Received	100 (99.2, 100.8)	0.0 (-0.1, 0.1)	-13.1 (-14.0, -12.1)	0.6 (0.3, 1.0)
Rate of HIV Tests Performed and Results Received	64.7 (56.8, 73.6)	-0.4 (-2.5, 1.8)	20.4 (1.5, 42.8)	-0.2 (-6.0, 5.9)
Rate of PLWH Treated with ART	83.2 (70.3, 98.1)	-1.1 (-3.8, 1.6)	12.8 (-9.1, 39.9)	-1.9 (-9.0, 5.7)
Ratio of Discharge Planning Visits per PLWH Released	1.6 (1.1, 2.7)	-1.8 (-7.8, 7.2)	11.4 (-45.9, 90.1)	-5.6 (-23.2, 22.6)

^a^ Probabilities modelled using segmented linear regression models

^b^ Refers to the rate in August 2019, the end of the first testing phase

^c^ Refers to the modelled change (%) per month during the pre‐transition period

^d^ Refers to the modelled change (%) immediately after the transition to LBAg/Ab testing compared to immediately before the transition

^e^ Refers to the modelled change (%) per month during the post-transition period

Regarding the receipt of ART, the rate of being a PLWH treated with ART on the first of the month was 83.2% (95% CI: 70.3, 98.1) in August 2019. After the transition to LBAg/Ab testing, the rate of being a PLWH treated with ART started at 93.8% (95% CI: -9.1, 39.9); however, the shift in the ART initiation rate across testing periods was not significant (Table 2). The rate of initiating ART did not change across the LBAg/Ab testing period. At baseline, the ratio of discharge planning visits per PLWH released was 1.6 (95% CI: 1.1, 2.7); this did not significantly change over the rPOC testing period (Table 2). After the transition to LBAg/Ab testing, the ratio of discharge planning visits per PLWH released was 1.8 (95% CI: 1.1, 2.7); however, this increase between testing periods was not statistically significant (Table 2). Additionally, the discharge planning ratio did not significantly change across the LBAg/Ab testing period.

## Discussion

This is the first study to describe changes in HIV testing parameters and elements of the HIV care cascade associated with a transition of routine HIV testing strategies at entry from third generation, rPOC testing to fourth generation, LBAg/Ab testing in a correctional setting. Analyzing HIV care and treatment outcomes in the D.C. DOC between January 2019 and January 2020, we determined that the transition from rPOC to LBAg/Ab testing contributed to a significant increase in the rate of HIV testing, a significant decrease in the rate of HIV results received, and a significant increase in the combined rate of HIV tests performed and HIV test results received. Additionally, there were upstream increases in the rate of PLWH receiving ART and the number of PLWH receiving discharge planning between time periods. We also determined that there was a statistically significant positive trend in the receipt of HIV results during the LBAg/Ab testing period, with the rate increasing by 0.6% each month following the transition.

The results of this study are important for several reasons. While HIV prevalence in the U.S. criminal justice system is up to ten times that of the general adult population, HIV testing remains inadequate in many correctional settings. Improving the testing strategy in correctional settings could begin or sustain linking PLWH to care [19–21]. This study contributes to a growing literature that the type of test performed is important, particularly in settings like jails where the median length of stay is 2–7 days [8]. Rapid POC testing requires only minutes for healthcare staff to perform and inform patients of results. We hypothesized that rPOC testing would result in more HIV tests performed; however, the ease of adding HIV testing to a panel of other laboratory tests routinely drawn may have led to an increase in HIV tests performed in the LBAg/Ab testing period.

Despite an increase in testing, we determined that the percentage of HIV test results received decreased from the rPOC to LBAg/Ab time period, even in a jail with a longer than average median length of stay [8]. This difference between testing periods was statistically significant in both the analysis where we assumed that 100% received rPOC test results at intake and the sensitivity analysis where we compared only the receipt of letters notifying residents of results of tests performed. The way in which LBAg/Ab testing might have resulted in a lower percentage of test results received among those tested is twofold: 1) incarcerated individuals may be discharged before their results return, 2) incarcerated individuals may not be stably housed to receive their results through mail after release. Fewer people receiving their test results represent a missed opportunity to inform an individual about their HIV status. Delays associated with receiving test results may have profound impacts, such as not initiating ART or not using barrier protection with sex. With increasing use of PrEP, provision of negative HIV test results may also be coupled with counseling for those who are at risk of HIV.

This study builds on previous work showing that the testing strategies implemented in jail settings matter. For example, an study of three large urban jails demonstrated six to seven-fold increases in the proportion of detainees who completed testing after rPOC testing began and led to success in identifying newly infected PLWH and proving care to PLWH while incarcerated [22]. At the Fulton County Jail in Atlanta, Georgia, a routine, opt-out, rapid HIV screening program was implemented for entrants in 2010. After this program was terminated in 2017 due to halted funding, HIV testing was limited to clinician-initiated conventional laboratory-based tests with up to a week turn-around for positive tests. The rapid screening program administered 1,420 tests/month and identified 89 (0.5%) new HIV infections a year [13] compared to the clinician-initiated program, which only administered 333 tests/month and identified 15 (0.4%) infections in 2018 with three patients with newly identified HIV leaving and never receiving test results [23]. The former strategy of routine screening resulted in an additional 74 new HIV diagnoses, 8.4 HIV transmissions averted, 45 Quality Adjusted Life Years gained over a year. It was also cost-saving to society when compared to the clinician-initiated program, which resulted in $3.7 million in additional costs to the healthcare system [23].

### Limitations

The generalizability of the finding that HIV testing increased with transition from rPOC to LBAg/Ab testing may be limited. Unlike most jails, the D.C. DOC offers a panel of laboratory tests to all entrants. Most jails have a length of stay between 2 and 7 days and most do not phlebotomize entrants routinely [15]. Therefore, further data are needed on the performance characteristics of existing HIV tests in additional detention facilities to define the optimal HIV testing strategy in U.S. jails. Moreover, whether a laboratory-based HIV test would be accepted by jail entrants who otherwise would not have a blood draw needs further study. The outcome of a strategy of combining the two tests, rPOC and laboratory-based testing, is also unknown. Lastly, rPOC technology continues to improve. An FDA-approved rPOC fourth generation Ag/Ab is now available. Combining the advantages of more sensitive screening withAg/Ab testing along with the speed of rPOC tests may maximize the viral detection of, and provision of test results to, all PLWH passing through jail [24]. Combining rPOC testing with a specimen sent to a laboratory will permit reflex testing to confirm the rapid test result.

## Conclusions

In a jail that offers phlebotomy-based laboratory testing on all entrants, we observed an increase in the HIV testing rate following a transition from rPOC to LBAg/Ab testing; however, rPOC testing averted the delays in receiving test results associated with LBAg/Ab testing in a jail. The transition from rPOC to LBAg/Ab generation testing demonstrated that each strategy has strengths in helping identify PLWH circulating through the correctional system. Additional research including cost-effectiveness studies should be performed to evaluate whether a rPOC test combined with a laboratory based screening test with a reflex confirmatory test could be the best strategy for screening for HIV in jail settings.

Maximizing the yield of HIV testing and provision of test results in detention facilities could promote rapid entry into care for those who newly test positive, rapid re-engagement for those whose positive status is confirmed but have fallen out of care, and new engagement into PrEP for those who test HIV-negative. Ending the HIV epidemic will need public health and correctional systems to collaboratively manage HIV in jails more purposively.

## References

[1] Maruschak LM. HIV in Prisons, 2015—Statistical Tables, Bureau of Justice Statistics, NCJ 250641. Available: https://bjs.ojp.gov/content/pub/pdf/hivp15st.pdf Accessed 19 August 2021.

[2] Minton TD, Zeng Z. Jail inmates mid-year 2015. Washington, DC: US Department of Justice, Office of Justice Programs, Bureau of Justice Statistics. NCJ 50394 Available: https://www.bjs.gov/content/pub/pdf/ji15.pdf. Accessed 19 August 2021.

[3] SpauldingAC, SealsRM, PageMJ, BrzozowskiAK, RhodesW, HammettTM. HIV/AIDS among inmates of, and releasees from, US correctional facilities, 2006: declining share of epidemic but persistent public health opportunity. *PLoS One*. 2009;11(4):e7558.10.1371/journal.pone.0007558PMC277128119907649

[4] DaileyAF, HootsBE, HallHI, et al. Vital Signs: Human Immunodeficiency Virus Testing and Diagnosis Delays—United States. *MMWR Morbidity and Mortality Weekly Report*. 2017;66(47):1300–1306. doi: 10.15585/mmwr.mm6647e1 29190267PMC5708685

[5] Centers for Disease Control and Prevention. Fact Sheet: Understanding the HIV Care Continuum. Atlanta: Centers for Disease Control and Prevention; 2018. Available: www.cdc.gov/hiv/pdf/library/factsheets/cdc-hiv- care-continuum.pdf. Accessed 21 August 2018.

[6] IrohPA, MayoH, NijhawanAE. The HIV Care Cascade before, during, and after incarceration: a systematic review and data synthesis. *Am J Public Health*. 2015;105.10.2105/AJPH.2015.302635PMC446339525973818

[7] Maruschak LM, Bronson J, Alper M. Medical Problems Reported by Prisoners: Survey of Prison Inmates, 2016. NCJ 252644. Available: https://bjs.ojp.gov/sites/g/files/xyckuh236/files/media/document/mprpspi16st.pdf Accessed: 19 August 2021. 2021.

[8] SpauldingAC, PerezSD, SealsRM, KavaseryR, HallmanM, WeissP. The diversity of release patterns for jail detainees: implications for public health interventions. *American Journal of Public Health*. 2011;101(Suppl 1):S347–S352.2203904210.2105/AJPH.2010.300004PMC3222492

[9] Zeng Z, Minton TD. Jail inmates in 2019. Bureau of Justice Statistics, March 2021, NCJ 255608. Available: https://bjs.ojp.gov/library/publications/jail-inmates-2019. Accessed 19 August 2021.

[10] Carlson AE. Prisoners in 2019. Bureau of Justice Statistics, October 2020, NCJ 255115. Available: https://bjs.ojp.gov/content/pub/pdf/p19.pdf. Accessed 19 August 2021.

[11] Kaeble D, Glaze L. Correctional Populations in the United States, 2015. Bureau of Justice Statistics. NCJ 250374. Available: https://www.bjs.gov/content/pub/pdf/cpus15.pdf. Accessed: 7 January 2017. 2016.

[12] BeckwithCG, Atunah-JayS, CohenJ, et al. Feasibility and acceptability of rapid HIV testing in jail. AIDS Patient Care and STDs. 2007;21(1):41–47. doi: 10.1089/apc.2006.006 17263656

[13] SpauldingAC, KimMJ, CorpeningKT, CarpenterT, WatlingtonP, BowdenCJ. Establishing an HIV Screening Program Led by Staff Nurses in a County Jail. *Journal of Public Health Management and Practice*. 2015.10.1097/PHH.0000000000000183PMC449287425427254

[14] PetersenJ, MonteiroM, DalalS, JhalaD. Reducing false-positive results with fourth-generation HIV testing at a Veterans Affairs Medical Center. Federal Practitioner. 2021;(38 No. 5). doi: 10.12788/fp.0125 34177233PMC8221825

[15] Centers for Disease Control and Prevention. *HIV testing implementation guidance for correctional settings*. 2009. Available: https://stacks.cdc.gov/view/cdc/5279/cdc_5279_DS1.pdf. Accessed 19 August 2021.

[16] Hutchinson AB, MacGowan R, Margolis A, Adee MG*, Bowden CJ, Spaulding AC. June 2019. Costs and Consequences of Eliminating a Routine HIV Screening Program in a High Prevalence Jail. PS 1–31, 41^st^ Annual Meeting of the Society for Medical Decision Making, Portland OR, October 20–23, 2019.

[17] United States Department of Justice. Office of Justice Programs. Bureau of Justice Statistics. Annual Survey of Jails, 2017. Inter-university Consortium for Political and Social Research [distributor], 2019-10-10. 10.3886/ICPSR37373.v1. Accessed 19 November 2019.

[18] The DC Department of Corrections. DC Department of Corrections Facts and Figures: June 2021. 2021. Available: https://doc.dc.gov/sites/default/files/dc/sites/doc/publication/attachments/DC%20Department%20of%20Corrections%20Facts%20and%20Figures%20June%202021.pdf. Accessed 19 August 2021.

[19] SolomonL, MontagueBT, BeckwithCG, et al. Survey finds that many prisons and jails have room to improve HIV testing and coordination of postrelease treatment. *Health Affairs*. 2014;33(3):434–442. doi: 10.1377/hlthaff.2013.1115 24590942PMC4028701

[20] ElkingtonKS, JaiswalJ, SpectorAY, et al. Can TasP Approaches Be Implemented in Correctional Settings?: A review of HIV testing and linkage to community HIV treatment programs. *J Health Care Poor Underserved*. 2016;27(2a):71–100. doi: 10.1353/hpu.2016.0047 27133513PMC5599929

[21] HerceME, HoffmannCJ, FieldingK, ToppSM, HauslerH, ChimoyiL, et al. Universal test-and-treat in Zambian and South African correctional facilities: a multisite prospective cohort study. The Lancet HIV. 2020 Dec 1;7(12):e807–16. doi: 10.1016/S2352-3018(20)30188-0 32763152

[22] BeckwithCG, NunnA, BaucomS, et al. Rapid HIV testing in large urban jails. American Journal of Public Health. 2012;102(S2). doi: 10.2105/AJPH.2011.300514 22401524PMC3477921

[23] Francis-GrahamS, EkekeNA, NelsonCA, et al. Understanding how, why, for whom, and under what circumstances opt-out blood-borne virus testing programmes work to increase test engagement and uptake within prison: a rapid-realist review. *BMC health services research*. 2019;19(1):152. doi: 10.1186/s12913-019-3970-z 30849986PMC6408812

[24] FDA Center for Biologics Evaluation and Research. Determine HIV-1/2 ag/ab combo. U.S. Food and Drug Administration. https://www.fda.gov/vaccines-blood-biologics/approved-blood-products/determine-hiv-12-agab-combo. Published January 31, 2022. Accessed December 16, 2022.

